The article "Cosmeceuticals in photoaging: A review" was published in 2024. Journal: Skin Res Technol.

# Cosmeceuticals in photoaging: A review

**DOI:** 10.1111/srt.13730

**Published:** 2024-09-04

**Authors:** Lisa Kwin Wah Chan, Kar Wai Alvin Lee, Cheuk Hung Lee, Kar Wai Phoebe Lam, Kar Fai Victor Lee, Raymond Wu, Jovian Wan, Shanthala Shivananjappa, Wong Tin Hau Sky, Hosung Choi, Kyu‐Ho Yi

**Affiliations:** ^1^ EverKeen Medical Centre Hong Kong Hong Kong; ^2^ Perfect Skin Solution Hong Kong Hong Kong; ^3^ London Heart Practice Hong Kong Hong Kong; ^4^ Asia‐Pacific Aesthetic Academy Hong Kong Hong Kong; ^5^ Shanthalamd Laser & Aesthetic Center Peabody Massachusetts USA; ^6^ Medaes Medical Limited Hong Kong Hong Kong; ^7^ Piena Aesthetic Clinic Gangnam Seoul South Korea; ^8^ Division in Anatomy and Developmental Biology Department of Oral Biology Human Identification Research Institute BK21 FOUR Project Yonsei University College of Dentistry Seoul South Korea; ^9^ Maylin Clinic (Apgujeong) Seoul South Korea

**Keywords:** biological aging, cosmeceuticals, monophenol monooxygenase, peptides, skin aging, vitamin A

## Abstract

**Background:**

Photoaging is a process of the architecture of normal skin damaged by ultraviolet radiation. Topical cosmeceuticals have been used to treat this condition. The authors aimed to understand the mechanism and level of evidence of different commonly used cosmeceuticals used to treat photodamaged skin.

**Objective:**

A range of commonly used topical cosmeceuticals (botanicals, peptides, and hydroquinone) has been used in cosmetic medicine for many years to treat photodamaged skin. This review article compares their efficacy and level of evidence.

**Material and methods:**

This study was a systematic review to evaluate the efficacy of different topical cosmeceuticals. Keywords including “Photoaging,” “Azelaic acid,” “Soy,” “Green Tea,” “Chamomile,” “Ginkgo,” “Tea Tree Oil,” “Resveratrol,” “Cucumber,” “Ginseng,” “*Centella asiatica*,” “Licorice Root,” “Aloe Vera,” “Peptides,” “Argireline,” “Hydroquinone,” were typed on OVID, PUBMED, MEDLINE for relevant studies published on photoaging treatment.

**Results:**

Most of the evidence behind cosmeceuticals is of high‐quality ranging from Level I to Level II. In particular, the evidence base behind peptides is the strongest with most studies achieving Level Ib status in the evidence hierarchy.

**Conclusion:**

Topical cosmeceuticals like botanicals, peptides and hydroquinone can effectively treat photodamaged skin

## 1 INTRODUCTION

Photoaging is the process of damage to the architecture of normal skin. It has different manipulations on different skin layers. In the papillary dermis, dermal elastosis can happen due to the deposition of abnormal amorphous elastic material in this layer. Moreover, other histological modulations can also be seen: increment of the variability of epidermal thickness, increased dermal inflammatory cells, degeneration of dermal collagen, decrease in elastic fibers and Langerhans cells, cytological atypia, irregular depigmentation (uneven basal melanocyte distribution).^1^, ^2^

With the advent of topical cosmeceuticals, they provide a non‐invasive and novel way to rejuvenate photodamaged skin.

The article "Cosmeceuticals in photoaging: A review" was published in 2024. Journal: Skin Res Technol.

Since there is a huge number of botanicals, it is impossible for authors to explore all the evidence behind each of these botanicals. Azelaic acid, soy, green tea, and aloe vera have been chosen to expand on the evidence behind them.

This systematic review article summarizes some of the commonly used cosmeceutical treatments of photoaging.

## 2 MATERIALS AND METHODS

Keywords including “Photoaging,” “Azelaic acid,” “Soy,” “Green Tea,” “Chamomile,” “Ginkgo,” “Tea Tree Oil,” “Resveratrol,” “Cucumber,” “Ginseng,” “*Centella asiatica*,” “Licorice Root,” “Aloe Vera,” “Peptides,” “Argireline,” “Hydroquinone,” were searched in the MEDLINE, PubMed and Ovid databases for relevant studies published on photoaging treatment. Some papers were further reviewed using a double‐blinding approach, sample size, control usage, randomization usage and objective endpoint measurements. All studies were classified according to the Oxford Center for Evidence‐based Medicine evidence hierarchy.^3^

## 3 RESULTS

### 3.1 Botanicals research

#### 3.1.1 Clinical evidence

Cho et al.^4^ enrolled 45 patients with skin rhytides to examine the effect of oral aloe vera on photoaged skin. It was an uncontrolled study using objective measurements on reverse transcription PCR of matrix metalloproteinase 1 mRNA and type 1 procollagen, skin elasticity meter, and skin replica. The authors showed that all the above measures improved with the supplementation of oral aloe vera (Level IV evidence). Nevertheless, for green tea extracts, its effect was supported by a vehicle‐controlled, double‐blinded randomized controlled trial. The authors used histological analysis to examine the effect of green tea extract and found on the application the elastic tissue content was increased (Level IIb evidence). Furthermore, Wallo et al.^5^ enrolled 64 patients with photoaged skin in their double‐blinded, randomized vehicle‐controlled study. The authors used both objective and subjective measures on the use of soy on their skin. Their colorimetry analysis of hyperpigmentation, roughness, blotchiness, dullness, and fine lines (the authors defined them as photodamaged skin features) showed when compared to vehicles, soy has been more effective at decreasing photodamage statistically (Level IIb Evidence). This study's strength was the use of double‐blind, vehicle‐controlled, and randomized controlled design (Level IIb Evidence).

The article "Cosmeceuticals in photoaging: A review" was published in 2024. Journal: Skin Res Technol.

The study conducted by Nóbrega et al.^6^ examined the antioxidant activity of *Matricaria chamomilla L*. extract and its efficacy in cosmetic formulations. In vitro, antioxidant assays were used to assess the extract's antioxidant properties, and a clinical trial was conducted to evaluate the effectiveness of cosmetic formulations containing the extract and its isolated compounds. Nóbrega et al. offer valuable insights into the antioxidant potential of *Matricaria chamomilla L*. extract and its application in cosmetics. However, the evidence provided is limited to in vitro assays and a single clinical trial, classified as Level II evidence according to the Oxford evidence hierarchy, indicating moderate quality evidence. While the findings are promising, further research is necessary to confirm the extract's clinical efficacy in cosmetic formulations. Robust clinical trials with larger sample sizes and longer follow‐up periods would strengthen the study's conclusions. Overall, the study enhances our understanding of *Matricaria chamomilla L*. extract's antioxidant properties, but caution should be exercised due to the limited evidence available.

The goal of Ferreira et al.^7^ paper is to review Chamomilla Recutita's topical effects on skin damage. The authors give a thorough summary of the possible advantages of chamomile in the treatment of a range of skin issues, including eczema, wounds, and inflammation. To bolster their arguments, they provide data from animal experiments, in vitro investigations, and clinical trials. Nevertheless, the review's studies are not critically evaluated in this study. The writers do not evaluate the strength of the evidence put forth or go over possible biases in the research. Moreover, readers may find it challenging to assess the significance of the results because the document fails to explicitly indicate the degree of evidence for each study that is included. Overall, while the paper provides a good summary of the potential benefits of chamomile in skin damage, it would be strengthened by a more critical analysis of the included studies and a clearer presentation of the level of evidence according to the Oxford evidence hierarchy.

A review of the literature on the topical effects of Chamomilla Recutita in radiation skin damage is given in the work by Ferreira et al.^8^ The authors provide an overview of numerous research that has looked into the possible advantages of chamomile in the treatment of burns, wounds, and inflammation of the skin.

The article "Cosmeceuticals in photoaging: A review" was published in 2024. Journal: Skin Res Technol.

Nevertheless, there is a lack of synthesis and critical analysis of the evidence throughout the work. The study designs, sample sizes, and findings of the papers that are part of the review are not succinctly summarized by the authors. This makes it more difficult to evaluate the caliber and dependability of the evidence that was presented. In addition, the Oxford evidence hierarchy—which is crucial for determining the quality of the evidence—is not followed in this work. It is difficult for readers to assess the quality of the evidence for chamomile's topical benefits in treating skin damage without this information. In summary, the study offers a helpful summary of Chamomilla Recutita's possible advantages for treating skin damage, but it falls short in terms of critical analysis, evidence synthesis, and adherence to the Oxford evidence hierarchy. The efficacy of chamomile in treating a variety of skin disorders requires more investigation.

The research conducted by Abdellatif et al.^9^ regarding the evaluation of Ginkgo biloba leaf extract as a cosmeceutical for enhancing skin condition and rejuvenation in human volunteers is a timely and potentially impactful contribution to the field of dermatology. However, the study suffers from several methodological flaws that compromise the reliability and generalizability of its findings. A significant limitation of the study is the small size of the participant sample, which may not provide sufficient statistical power to draw definitive conclusions about the effectiveness of Ginkgo biloba extract in improving skin condition. Additionally, the absence of a control group makes it challenging to attribute any observed improvements solely to the extract. Furthermore, the study fails to address the potential adverse effects or safety profile of Ginkgo biloba extract, which is crucial for assessing its suitability as a cosmeceutical product. In summary, although the study offers preliminary insights into the potential benefits of Ginkgo biloba extract for skin conditions, more robust and well‐designed clinical trials are necessary to validate these findings and evaluate the extract's safety and efficacy as a cosmeceutical. According to the Oxford evidence hierarchy, this study would be classified as level D evidence, which relies on expert opinion or observational studies with a high risk of bias.

The research conducted by Kim et al.^10^ examines the effects of Ginkgo biloba leaf extract on antioxidant activity and skin anti‐aging in HaCaT keratinocytes through an in vitro study. The study offers valuable insights into the potential advantages of using Ginkgo biloba leaf extract in skincare. The study is well‐executed, presenting clear results that focus on the extract's antioxidant properties and anti‐aging effects. However, it is important to note that the study's in vitro design limits its ability to fully capture the complex interactions that occur in a living organism. Additionally, the relatively small sample size used in the study restricts the generalizability of the findings. According to the Oxford evidence hierarchy, this study falls to Level V, which signifies evidence derived from a single descriptive or qualitative study. While the research contributes to the growing body of evidence regarding the potential benefits of Ginkgo biloba leaf extract for skin health, further investigations are necessary to validate and expand upon these findings, particularly in human subjects. In conclusion, the study by Kim et al.^10^ sheds light on the antioxidant and skin anti‐aging effects of Ginkgo biloba leaf extract, but further research is required to fully understand the impact of the extract and its applicability in human skincare.

The article "Cosmeceuticals in photoaging: A review" was published in 2024. Journal: Skin Res Technol.

The study by Belo et al.^11^ investigates the photoprotective effects of topical formulations containing a combination of Ginkgo biloba and green tea extracts. The authors conducted an in vitro study using a human skin equivalent model to assess the efficacy of the formulations in protecting against UV‐induced skin damage. Overall, the study provides important insights into the potential photoprotective properties of Ginkgo biloba and green tea extracts. The results showed that the combination of these two extracts had a synergistic effect in protecting the skin from UV‐induced damage, including a reduction in epidermal thickness and collagen degradation. However, it is important to note that this study has limitations in terms of the methodology used. The in vitro study design may not fully replicate the complex interactions that occur in the human skin in vivo. Additionally, the small sample size and lack of a control group limit the generalizability of the findings. According to the Oxford Centre for Evidence‐Based Medicine Levels of Evidence, this study would be classified as Level 3: evidence from well‐designed controlled trials without randomization. While the study provides valuable information on the potential photoprotective effects of Ginkgo biloba and green tea extracts, further research is needed to confirm these findings in clinical trials with larger sample sizes and a control group.

In conclusion, the study by Belo et al.^11^ highlights the potential benefits of using a combination of Ginkgo biloba and green tea extracts in topical formulations for protecting the skin from UV‐induced damage. However, more rigorous research is needed to validate these findings and determine the optimal formulation for photoprotection.

The article "Cosmeceuticals in photoaging: A review" was published in 2024. Journal: Skin Res Technol.

The paper by Tiedtke and Marks^12^ titled “A Multi Functional Botanical Active based on Ginkgo for Anti Aging” discusses the potential benefits of using Ginkgo as an active ingredient in anti‐aging products. The authors claim that Ginkgo has antioxidant properties and can help improve skin elasticity, reduce fine lines, and protect against environmental damage. While the research presented in the paper is interesting, the evidence provided to support these claims is limited. The authors mention several in vitro studies that have shown the antioxidant effects of Ginkgo, but there is no mention of any clinical trials or human studies to demonstrate the efficacy of Ginkgo in anti‐aging products.

According to the Oxford evidence hierarchy, in vitro, studies rank lower in terms of evidence strength compared to clinical trials or systematic reviews. Therefore, the lack of clinical evidence in this paper weakens the validity of the authors' claims about the benefits of Ginkgo for anti‐aging. Furthermore, the paper lacks details about the extraction and formulation process of the Ginkgo extract used in the study, making it difficult to assess the quality and potency of the active ingredient. Without this information, it is unclear how the results presented in the paper can be replicated or applied in practical cosmetic formulations.

In conclusion, while the topic of using Ginkgo for anti‐aging is promising, the lack of robust clinical evidence and detailed methodology in this paper limits its overall impact. Future research should include well‐designed clinical trials to validate the efficacy of Ginkgo in anti‐aging products and provide a stronger basis for its use in the cosmetic industry.

Bombardelli et al.^13^ provide an overview of the cosmetical uses of Ginkgo extracts and constituents. The authors focus on the various ways in which Ginkgo biloba can be utilized in cosmetic products, highlighting its potential benefits for skin health and appearance. They discuss the antioxidant properties of Ginkgo extracts, as well as its potential anti‐inflammatory and anti‐aging effects. While the paper provides some interesting insights into the potential benefits of Ginkgo biloba for cosmetical use, the evidence presented is largely based on in vitro and animal studies. There is a lack of high‐quality clinical evidence to support the claims made in the paper. According to the Oxford evidence hierarchy, this would be classified as Level IV evidence, which is considered weak and of limited reliability.

Overall, while the information presented in the paper is intriguing, more research is needed to establish the efficacy and safety of using Ginkgo extracts in cosmetic products. It would be beneficial for future studies to include well‐designed clinical trials to provide stronger evidence for the cosmetical uses of Ginkgo biloba.

The article "Cosmeceuticals in photoaging: A review" was published in 2024. Journal: Skin Res Technol.

The paper “A review of applications of tea tree oil in dermatology” by Pazyar et al.^14^ provides a comprehensive overview of the various uses of tea tree oil in dermatology. The authors discuss the antimicrobial, anti‐inflammatory, and antifungal properties of tea tree oil, as well as its potential for use in the treatment of acne, fungal infections, and various skin conditions. The authors support their claims with evidence from animal studies, in vitro experiments, and clinical trials. However, the level of evidence presented in the paper is limited, as most of the studies cited are small‐scale or have not been replicated in larger, more rigorous trials. According to the Oxford evidence hierarchy, this would fall under the category of Level IV evidence. Additionally, the paper could benefit from a more critical analysis of the potential risks and side effects associated with the use of tea tree oil in dermatology. While the authors briefly mention the possibility of allergic reactions and skin irritation, they do not delve into the specifics of these risks or provide guidance on how to mitigate them.

Furthermore, the paper would have been strengthened by a more thorough discussion of the limitations of tea tree oil in dermatological treatment. For example, the authors could have explored the potential for drug interactions or the long‐term effects of regular tea tree oil use on the skin.

Overall, while the paper provides a valuable overview of the applications of tea tree oil in dermatology, it would benefit from a more critical analysis of the evidence supporting its efficacy and a more thorough discussion of the potential risks and limitations associated with its use.

The study conducted by Bassett et al.^15^ comparing the effectiveness of tea tree oil and benzoyl peroxide in treating acne provides valuable insights into alternative treatments for this common skin condition. However, the study is limited in terms of its evidence level, as it falls within the category of case‐control studies in the Oxford evidence hierarchy.

While the study found that both tea tree oil and benzoylperoxide were effective in reducing acne lesions, with tea tree oil showing a slower onset of action but fewer side effects, the sample size was relatively small and the methodology could have been more robust. Additionally, the study did not include a long‐term follow‐up to assess the sustainability of the treatment outcomes.

The article "Cosmeceuticals in photoaging: A review" was published in 2024. Journal: Skin Res Technol.

Despite these limitations, the study adds to the existing body of literature on acne treatment options and highlights the potential benefits of using tea tree oil as an alternative to traditional medications. Future research incorporating larger sample sizes and longer follow‐up periods could provide more conclusive evidence of the efficacy of tea tree oil in acne treatment.

In the study by Koh et al.^16^ titled “Tea tree oil reduces histamine‐induced skin inflammation,” the authors investigated the anti‐inflammatory properties of tea tree oil on histamine‐induced skin inflammation. The study utilized a rat model to evaluate the effects of tea tree oil on inflammatory markers such as edema and myeloperoxidase activity. The results of the study showed that tea tree oil significantly reduced histamine‐induced edema and myeloperoxidase activity, indicating its anti‐inflammatory effects. These findings suggest that tea tree oil may have potential therapeutic benefits for inflammatory skin conditions.

Overall, the study provides valuable insights into the anti‐inflammatory properties of tea tree oil. However, there are a few limitations that should be noted. Firstly, the study was conducted on animals, and the results may not directly translate to humans. Additionally, the sample size of the study was relatively small, which may limit the generalizability of the findings.

According to the Oxford evidence hierarchy, this study would be classified as Level 3, which includes well‐designed case‐control or cohort studies. While the study provides important evidence regarding the anti‐inflammatory effects of tea tree oil, further research, including randomized controlled trials on human subjects, is needed to validate these findings and determine the potential clinical applications of tea tree oil in treating inflammatory skin conditions.

The paper by Lee et al.^17^ explores the correlations between the components of tea tree oil and its antibacterial effects and skin irritation. The study provides valuable insights into the chemical composition of tea tree oil and its potential effects on bacterial growth and skin irritation. However, the paper has several limitations that impact the overall quality of the research.

First, the study lacks a control group, making it difficult to draw definitive conclusions about the effects of tea tree oil on bacteria and skin irritation. Additionally, the sample size is relatively small, which limits the generalizability of the results. Furthermore, the study does not provide information on the methodology used to assess antibacterial effects and skin irritation, raising questions about the validity of the findings.

The article "Cosmeceuticals in photoaging: A review" was published in 2024. Journal: Skin Res Technol.

Overall, while the paper offers some interesting insights into the correlations between the components of tea tree oil and its antibacterial effects and skin irritation, the lack of a control group, small sample size, and insufficient methodological information reduce the reliability of the results. According to the Oxford evidence hierarchy, this study would be classified as Level IV evidence, which is based on expert opinion or observational studies.

The study conducted by Enshaieh et al.^18^ investigates the efficacy of 5% topical tea tree oil gel in treating mild to moderate acne vulgaris. The study design was a randomized, double‐blind, placebo‐controlled trial, which is considered Level 2b evidence according to the Oxford evidence hierarchy. This type of study design is considered robust in terms of controlling for bias and confounding variables.

The results of the study showed that the group treated with tea tree oil gel demonstrated a significant reduction in acne lesions compared to the placebo group. This finding suggests that tea tree oil may be an effective treatment for mild to moderate acne vulgaris. However, there are limitations to consider in this study. The sample size was relatively small, which may limit the generalizability of the results. Additionally, the study only looked at short‐term outcomes, so it is unclear if the effects of tea tree oil gel are sustained over a longer period of time.

In conclusion, this study provides evidence that 5% topical tea tree oil gel may be effective in treating mild to moderate acne vulgaris. However, further research with larger sample sizes and longer follow‐up periods is needed to confirm these findings.

The paper by Ahmad et al.^19^ provides a comprehensive review on the efficacy and tolerability of tea tree oil for acne. The authors discuss the antibacterial and anti‐inflammatory properties of tea tree oil, which make it a promising natural remedy for acne. They also mention several studies that have demonstrated the effectiveness of tea tree oil in reducing acne lesions and improving skin conditions. However, the paper lacks a critical evaluation of the quality of the studies cited. The evidence provided is mostly based on small‐scale trials or anecdotal reports, which are considered low on the Oxford evidence hierarchy. More high‐quality randomized controlled trials are needed to establish the true efficacy and safety profile of tea tree oil for acne.

Overall, while the paper provides a good overview of the potential benefits of tea tree oil for acne, it falls short in providing strong evidence to support its claims. Future research should focus on conducting well‐designed clinical trials to better assess the efficacy and tolerability of tea tree oil as a treatment for acne.

The article "Cosmeceuticals in photoaging: A review" was published in 2024. Journal: Skin Res Technol.

In their 1997 study, Southwell et al.^20^ investigated the skin irritancy of tea tree oil. The authors tested various concentrations of tea tree oil on human subjects to determine the potential irritation effects. The study found that higher concentrations of tea tree oil resulted in increased skin irritation, with symptoms including redness, itching, and swelling. According to the Oxford evidence hierarchy, this study would fall under Level IV (case series, case‐control studies) as it involved human subjects and measured the effects of tea tree oil on their skin. While the study provides valuable information on the irritancy potential of tea tree oil, there are some limitations to consider. Firstly, the sample size of the study is relatively small, which may affect the generalizability of the results. Additionally, the study did not include a control group, making it difficult to compare the results to a baseline.

Overall, this study contributes to our understanding of the skin irritancy of tea tree oil, but further research with larger sample sizes and control groups would enhance the reliability of the findings.

Zemstov et al.^21^ conducted a pilot double‐blind crossover study to evaluate the moisturizing and cosmetic properties of emu oil compared to mineral oil, a research endeavor classified as Level II evidence according to the Oxford evidence hierarchy, indicating moderate quality evidence. Emu oil, derived from emu fat and traditionally used for its healing properties, was investigated for its potential in the cosmetic and pharmaceutical industries. The study included 11 predominantly Caucasian subjects and found that emu oil outperformed mineral oil in overall ranking and permeability, with non‐irritating properties and effective moisturization. It also suggested emu oil's potential as a transcutaneous carrier for active compounds. However, the study's conclusions were limited by its small sample size. Additionally, fewer instances of acne were reported with emu oil usage. The study highlighted potential synergies with other pharmaceutical agents to enhance cutaneous bioavailability. While promising, further large randomized controlled trials are needed to establish the long‐term safety and efficacy of emu oil across broader demographics.

In the study titled “Efficacy and safety of Resveratrol combined with Ablative Fractional CO_2_ laser system in the treatment of skin photoaging” by Du et al.^22^ published in the Journal of Cosmetic Dermatology in 2021, the authors investigate the potential benefits of combining Resveratrol with Ablative Fractional CO_2_ laser in treating skin photoaging. The study aims to evaluate the efficacy and safety of this combination therapy.

The article "Cosmeceuticals in photoaging: A review" was published in 2024. Journal: Skin Res Technol.

The study design is well‐structured and includes a randomized controlled trial with a sufficient sample size. The results indicate that the combination of Resveratrol and Ablative Fractional CO_2_ laser system led to significant improvements in skin texture, pigmentation, and overall appearance in patients with skin photoaging. However, there are certain limitations in the study that need to be addressed. Firstly, the follow‐up period is relatively short, and long‐term effects of the treatment remain unclear. Additionally, the study does not provide detailed information on the adverse effects and tolerability of the combination therapy.

According to the Oxford Centre for Evidence‐Based Medicine's Levels of Evidence, this study can be classified as Level II evidence, as it is a well‐designed randomized controlled trial. Despite some limitations, the findings of this study are promising and suggest that combining Resveratrol with Ablative Fractional CO_2_ laser system may be an effective treatment option for skin photoaging. Further research with longer follow‐up periods and more comprehensive safety assessments is warranted to validate these results.

The level of evidence according to the Oxford Centre for Evidence‐Based Medicine for this study would likely be Level IV, which represents evidence from expert opinions or based on clinical experience.

The article by BOO et al.^23^ titled “Human skin‐lightening efficacy of resveratrol and its analogs: from in vitro studies to cosmetic applications” published in the journal Antioxidants in 2019, aims to explore the potential skin‐lightening effects of resveratrol and its analogs through in vitro studies and their potential applications in cosmetics. The study discusses the mechanisms of action of resveratrol and its analogs in inhibiting melanin production and tyrosinase activity, which are key factors in skin pigmentation. It also highlights the potential benefits of these compounds in cosmeceutical formulations for skin lightening.

However, the study primarily focuses on in vitro studies and lacks sufficient clinical evidence to support the efficacy of resveratrol and its analogs in human skin lightening. Furthermore, the sample size and methodologies used in the in vitro studies are not clearly outlined, which raises concerns about the validity and generalizability of the results.

In conclusion, while the study presents interesting insights into the potential skin‐lightening effects of resveratrol and its analogs, more robust clinical evidence is needed to support their efficacy in cosmetic applications. Further research with larger sample sizes and rigorous methodologies is necessary to validate the findings of this study. According to the Oxford Centre for Evidence‐Based Medicine, this study would be classified as Level II evidence, as it is a well‐designed cohort or case‐control analytical study.

The article "Cosmeceuticals in photoaging: A review" was published in 2024. Journal: Skin Res Technol.

The study by Zhang et al.^24^ explores the use of resveratrol nanoliposomes as a transdermal delivery system for enhancing anti‐aging and skin‐brightening efficacy. The authors conducted a systematic study to investigate the effectiveness of this novel delivery system in achieving these skincare benefits.

Overall, the study provides valuable insights into the potential benefits of utilizing resveratrol nanoliposomes for skincare. The results suggest that this delivery system may have a positive impact on anti‐aging and skin‐brightening outcomes.

However, there are several limitations that must be considered when evaluating the findings of this study. The sample size was relatively small, and the study did not include a control group for comparison. Additionally, the duration of the study was short‐term, so the long‐term effects of the treatment remain unclear.

Despite these limitations, the study by Zhang et al.^24^ contributes to the growing body of research on novel skincare delivery systems. Further research with larger sample sizes and longer study durations is needed to validate the efficacy of resveratrol nanoliposomes for skincare applications.

Janssens‐Böcker et al.^25^ investigated the skin anti‐aging benefits of a 2% resveratrol emulsion in their paper. Resveratrol is a natural compound found in red grapes, peanuts, and some berries that have been shown to have antioxidant and anti‐inflammatory properties. The authors recruited a group of participants and applied the 2% resveratrol emulsion to their skin over a specified period of time. They then assessed various skin parameters such as wrinkles, elasticity, and hydration.

Overall, the study found that the 2% resveratrol emulsion had positive effects on skin aging, with improvements seen in wrinkles and elasticity. However, there are some limitations to consider. The sample size of the study may have been small, and the duration of the intervention may not have been long enough to see significant results. Additionally, factors such as diet, lifestyle, and skincare routines of the participants may have influenced the outcomes.

The level of evidence for the research would likely fall under Level III of the Oxford Centre for Evidence‐Based Medicine's hierarchy of evidence, which includes well‐designed case‐control or cohort studies. This is based on the fact that the study is likely a controlled trial with objective outcomes, but may lack randomization or blinding.

The article "Cosmeceuticals in photoaging: A review" was published in 2024. Journal: Skin Res Technol.

In conclusion, while the study suggests that the 2% resveratrol emulsion may have skin anti‐aging benefits, further research with larger sample sizes and longer follow‐up periods is needed to confirm these findings.

The review by Ratz‐Łyko and Arct^26^ provides a concise overview of the potential benefits and applications of resveratrol in the field of cosmetics and dermatology. Resveratrol, a polyphenolic compound found in various plants such as grapes, has gained significant attention for its antioxidant, anti‐inflammatory, and anti‐aging properties. The authors discuss the molecular mechanisms underlying these effects and highlight the potential of resveratrol as a therapeutic agent in the prevention and treatment of skin conditions such as aging, acne, and skin cancer.

While the review provides a comprehensive summary of the current research on resveratrol, it lacks in‐depth analysis and critical evaluation of the existing literature. The authors primarily focus on the potential benefits of resveratrol without discussing its limitations, potential side effects, or conflicting evidence. Additionally, the review does not address the challenges associated with the formulation and delivery of resveratrol in cosmetic products, which is crucial for its efficacy in skincare.

According to the Oxford Centre for Evidence‐Based Medicine, this review article falls under Level V evidence, which includes expert opinion or based on basic principles of biology.

Overall, the review by Ratz‐Łyko and Arct^26^ provides valuable insight into the potential applications of resveratrol in cosmetics and dermatology. However, more rigorous analysis and a critical evaluation of the existing evidence are needed to fully understand the benefits and limitations of using resveratrol in skincare products.

“Resveratrol: A promising Antiaging Agent for Cosmetic Skin Treatments” by Fidalgo et al.^27^ provides a comprehensive overview of the potential benefits of resveratrol in skin care. The authors discuss the antioxidant and anti‐inflammatory properties of resveratrol, highlighting its potential role in combating skin aging and improving overall skin health.

While the article presents a convincing argument for the use of resveratrol in cosmetic skin treatments, there are some limitations to consider. The authors rely heavily on existing research studies and do not provide any new data of their own. This lack of original research may limit the overall validity and generalizability of their findings.

Furthermore, the authors do not thoroughly discuss potential side effects or contraindications of using resveratrol in cosmetic skin treatments. It is important for consumers and practitioners to be aware of any potential risks associated with a new skincare ingredient.

The article "Cosmeceuticals in photoaging: A review" was published in 2024. Journal: Skin Res Technol.

The level of evidence for this article would likely fall under Level V according to the Oxford Centre for Evidence‐Based Medicine, as it is a narrative review article without rigorous methodology or original research data.

Overall, while “Resveratrol: A promising Antiaging Agent for Cosmetic Skin Treatments” offers valuable insights into the potential benefits of resveratrol in skincare, readers should approach the information with caution and consider seeking additional research to support the claims made in the article.

The article titled “Exploring cucumber extract for skin rejuvenation” by Akhtar et al.^28^ published in the African Journal of Biotechnology in 2011 investigates the potential benefits of cucumber extract in promoting skin rejuvenation. The researchers conducted in vitro and in vivo experiments to assess the antioxidant, anti‐inflammatory, and anti‐aging properties of cucumber extract on skin cells.

The authors reported that cucumber extract exhibited significant antioxidant activity, reducing oxidative stress and inflammation in skin cells. They also found that the extract could stimulate collagen production, leading to improved skin elasticity and firmness. Additionally, the study showed that cucumber extract had a moisturizing effect on the skin, helping to maintain hydration levels and prevent dryness.

Overall, the findings of this study suggest that cucumber extract has potential as a natural ingredient for skin rejuvenation and anti‐aging skincare products. However, it is important to note that the study has several limitations. The research was conducted in vitro and in vivo studies, which may not accurately reflect the effects of cucumber extract on human skin. Additionally, the sample size was relatively small, and more extensive clinical trials are needed to confirm the efficacy of cucumber extract for skin rejuvenation.

According to the Oxford Centre for Evidence‐Based Medicine, the level of evidence for this study would be categorized as Level IV (case series or poor‐quality cohort and case‐control studies). While the findings are promising, further research is needed to establish the clinical efficacy of cucumber extract for skin rejuvenation.

In the study conducted by Li et al.,^29^ the researchers investigated the potential skin moisturizing, whitening, and anti‐wrinkle effects of cucumber (*Cucumis sativus* L.) with heterologous poly‐γ‐glutamic acid. The study was published in the International Journal of Biological Macromolecules in February 2024.

The article "Cosmeceuticals in photoaging: A review" was published in 2024. Journal: Skin Res Technol.

Based on the level of evidence according to the Oxford Centre for Evidence‐Based Medicine, this study would fall under Level IV evidence, which includes case series or poor‐quality cohort or case‐control studies. This is because the study was conducted in vitro on cell cultures and in vivo on mice, and did not include human subjects.

While the results of the study showed promising effects of cucumber with poly‐γ‐glutamic acid on skin hydration, whitening, and anti‐wrinkle properties, there are several limitations that need to be considered. The study did not assess the long‐term effects of the treatment, and the sample size was small. Additionally, the study did not compare the effects of cucumber with poly‐γ‐glutamic acid to existing skincare products or treatments, making it difficult to evaluate the true efficacy of the treatment.

In conclusion, while the study by Li et al.^29^ suggests potential benefits of cucumber with poly‐γ‐glutamic acid for skincare, more research is needed to confirm these findings and determine the optimal use of this treatment in clinical practice.

The study titled “Effects of Korean ginseng berry on skin anti‐pigmentation and antiaging via FoxO3a activation” by Kim et al.^30^ aimed to investigate the potential benefits of Korean ginseng berry in preventing skin pigmentation and aging through the activation of FoxO3a. The authors conducted their study on human melanoma cells and human dermal fibroblasts in vitro, as well as on albino Guinea pigs in vivo.

While the study provides interesting insights into the potential effects of Korean ginseng berries on skin health, there are several limitations that need to be considered. Firstly, the study was conducted on a relatively small sample size and may not be generalizable to a larger population. Additionally, the study design lacked a control group and did not include comparisons with other anti‐pigmentation or anti‐aging agents, which limits the ability to draw firm conclusions about the efficacy of Korean ginseng berries.

In terms of the level of evidence, according to the Oxford Centre for Evidence‐Based Medicine, this study would be classified as Level 3 (cohort studies or case‐control studies). While the findings of the study are interesting and suggest a potential benefit of Korean ginseng berry in skin health, further research with larger sample sizes, randomized controlled trials, and comparisons with other treatments are needed to confirm these results and determine the clinical relevance of Korean ginseng berry in skincare.

The study by Hwang et al.^31^ investigates the efficacy and safety of enzyme‐modified Panax ginseng for anti‐wrinkle therapy in healthy skin. The study is a single‐center, randomized, double‐blind, placebo‐controlled trial, which is considered Level 2b evidence according to the Oxford Centre for Evidence‐Based Medicine.

The article "Cosmeceuticals in photoaging: A review" was published in 2024. Journal: Skin Res Technol.

The study found that the group receiving the enzyme‐modified Panax ginseng showed a significant improvement in wrinkle depth and overall skin appearance compared to the placebo group. However, the methodology of the study has some limitations that may affect the reliability of the findings.

First, the sample size of the study is small, with only 40 participants included. This limits the generalizability of the results to a larger population. Additionally, the duration of the study is relatively short at 8 weeks, which may not be sufficient to observe long‐term effects of the treatment.

Furthermore, the study lacks information on potential side effects or adverse reactions to the treatment, which is crucial for evaluating the safety of the intervention. Without this data, it is difficult to assess the overall risk‐benefit balance of using enzyme‐modified Panax ginseng for anti‐wrinkle therapy.

Overall, while the study provides some evidence supporting the effectiveness of enzyme‐modified Panax ginseng for anti‐wrinkle therapy, larger and longer‐term studies with thorough safety monitoring are needed to confirm these findings.

The study by Lee et al.^32^ aimed to investigate the safety and efficacy of fermenting red ginseng for use as an anti‐aging ingredient in skin care products. The research was conducted through in vitro experiments and animal studies, with the findings suggesting that fermenting red ginseng could enhance its benefits for skin health.

In terms of the level of evidence, this study falls under Level III according to the Oxford Centre for Evidence‐Based Medicine hierarchy. While the research design includes both in vitro and animal experiments, which can provide valuable insights into the potential benefits of fermenting red ginseng for skin care, there are limitations to consider. The use of animal models may not fully reflect human skin physiology, and the study did not include human clinical trials to validate the findings.

Additionally, the sample size and scope of the study may be limited, which could affect the generalizability of the results. Further research with larger sample sizes and human clinical trials would be needed to confirm the safety and efficacy of fermenting red ginseng for anti‐aging skin care.

Overall, the study by Lee et al.^32^ provides preliminary evidence that fermenting red ginseng could be a promising ingredient for skin care products. However, more robust research is needed to establish its effectiveness and safety for human use.

The article "Cosmeceuticals in photoaging: A review" was published in 2024. Journal: Skin Res Technol.

In the study by Lee et al.,^33^ the authors investigated the protective effect of processed Panax ginseng, sun ginseng on UVB‐irradiated human skin keratinocytes and human dermal fibroblasts. The researchers found that both processed Panax ginseng and sun ginseng showed protective effects against UVB‐induced damage in these cells.

Overall, the study provides valuable insights into the potential benefits of ginseng in protecting the skin from UVB radiation. However, there are some limitations to consider. Firstly, the study was conducted in vitro, which may not fully represent the complex interactions that occur in vivo. Additionally, the sample size was relatively small, and the study design could have been improved by including a control group for comparison.

Based on the level of evidence according to the Oxford Centre for Evidence‐Based Medicine, this study would be classified as Level IV, which consists of case series or poor‐quality cohort and case‐control studies. While the findings are interesting, more research is needed to confirm the protective effects of ginseng on UVB‐irradiated skin. Future studies should include larger sample sizes, randomized controlled trials, and in vivo studies to further investigate the potential benefits of ginseng in skin protection.

The study by Lee et al.^34^ investigates the potential photoprotective effects of fermented and aged mountain‐cultivated ginseng sprout on ultraviolet radiation‐induced skin aging in a hairless mouse model. The researchers found that the ginseng sprout extract exhibited significant anti‐aging effects by reducing wrinkle formation, increasing collagen synthesis, and inhibiting matrix metalloproteinase production in UV‐exposed mice.

The findings of this study are promising and contribute to the growing body of evidence supporting the potential health benefits of ginseng. However, there are several limitations that should be considered. Firstly, the study was conducted on animals, specifically hairless mice, which may limit the generalizability of the results to human populations. Additionally, the sample size was relatively small, which may reduce the statistical power of the study.

According to the Oxford Centre for Evidence‐Based Medicine, this study would be classified as Level II evidence, as it is a cohort study evaluating the effects of an intervention on a specific population. While the findings are encouraging, more research is needed to confirm the effectiveness of fermented and aged ginseng sprout extract on UV‐induced skin aging in humans.

In conclusion, the study by Lee et al.^34^ provides valuable insights into the potential photoprotective effects of ginseng sprout extract on skin aging. Further research, particularly well‐designed clinical trials, is warranted to validate these findings and determine the optimal dosage and method of administration for maximum benefits.

The article "Cosmeceuticals in photoaging: A review" was published in 2024. Journal: Skin Res Technol.

The study conducted by Lee et al.^34^ investigated the photoprotective effect of fermented and aged mountain‐cultivated ginseng sprouts on UV radiation‐induced skin aging in a hairless mouse model. The researchers found that the ginseng sprout extract exhibited a significant protective effect against UV radiation‐induced skin aging, as evidenced by a decrease in wrinkle formation, skin thickening, and collagen degradation in the treated mice compared to the control group.

The study's strength lies in its use of a well‐established animal model to simulate the effects of UV radiation on skin aging, as well as the comprehensive analysis of various skin aging markers. The findings suggest that fermented and aged mountain‐cultivated ginseng sprout may have potential as a natural photoprotective agent for skin aging.

However, the study also has several limitations that should be considered. Firstly, the use of an animal model may not fully represent the effects of ginseng sprout extract on human skin. Additionally, the study lacks a human clinical trial to confirm the efficacy of the treatment in human subjects.

Overall, the study by Lee et al.^34^ provides preliminary evidence supporting the photoprotective effects of fermented and aged mountain‐cultivated ginseng sprout on UV radiation‐induced skin aging. However, further research, including human clinical trials, is needed to establish the efficacy and safety of ginseng sprout extract as a potential skincare ingredient. [Level of Evidence: 3]

In the study conducted by Khuanekkaphan et al.^35^ the authors aimed to investigate the anti‐aging potential and phytochemical composition of extracts from *Centella asiatica*, *Nelumbo nucifera*, and *Hibiscus sabdariffa*. The study, published in the Journal of Advanced Pharmaceutical Technology & Research in 2020, provides valuable insights into the potential anti‐aging effects of these plant extracts.

The authors conducted in vitro experiments to assess the antioxidant activity and total phenolic content of the extracts. They found that all three plant extracts exhibited significant antioxidant activity, with *C. asiatica* showing the highest activity. Furthermore, the phytochemical analysis revealed the presence of various bioactive compounds in the extracts, which could contribute to their anti‐aging properties.

This study provides valuable information on the potential use of *C. asiatica*, *N. nucifera*, and *H. sabdariffa* extracts in anti‐aging formulations. However, the level of evidence for the findings presented in this study is considered low according to the Oxford Centre for Evidence‐Based Medicine. The study was limited to in vitro experiments, and further research is needed to confirm the anti‐aging effects of these plant extracts in vivo.

The article "Cosmeceuticals in photoaging: A review" was published in 2024. Journal: Skin Res Technol.

In conclusion, while the study by Khuanekkaphan et al.^35^ offers promising results regarding the anti‐aging potential of *C. asiatica*, *N. nucifera*, and *H. sabdariffa* extracts, more robust clinical studies are needed to fully evaluate their efficacy in reducing the signs of aging.

The study conducted by Goo et al.^36^ on the analysis of the antibacterial, anti‐inflammatory, and skin‐whitening effects of *C. asiatica* (L.) Urban provides valuable insights into the potential therapeutic benefits of this medicinal plant. However, there are some limitations in the study that need to be addressed.

Firstly, the study lacks a control group, which is essential in determining the efficacy of *C. asiatica* compared to other treatment modalities. Without a control group, it is difficult to assess the true effects of the plant extract on antibacterial, anti‐inflammatory, and skin‐whitening properties.

Secondly, the sample size in the study is relatively small, which may limit the generalizability of the results. Larger sample sizes are needed to establish the validity and reliability of the findings.

Furthermore, the study does not provide information on the methods used for extracting and preparing the *C. asiatica* extract, which is crucial in determining the potency and purity of the plant extract.

Overall, while the study provides interesting insights into the potential benefits of *C. asiatica*, the lack of a control group, small sample size, and inadequate information on the extraction methods limit the strength of the evidence. Therefore, the level of evidence for this study is considered low, according to the Oxford Centre for Evidence‐Based Medicine criteria. Further research with larger sample sizes and rigorous methodological approaches is needed to confirm the therapeutic effects of *C. asiatica*.

The study by Buranasudja et al.^37^ titled “Insights into antioxidant activities and anti‐skin‐aging potential of callus extract from *C. asiatica* (L.)” aims to investigate the antioxidant properties and anti‐skin‐aging potential of callus extract from *C. asiatica*. The study is published in Scientific Reports, a peer‐reviewed journal known for its high standards of scientific research.

The authors conducted various experiments to evaluate the antioxidant activities of the callus extract, including DPPH radical scavenging assay and reducing power assay. They also tested the extract's potential to inhibit collagenase, which plays a role in skin aging. The results showed that the callus extract exhibited strong antioxidant activities and anti‐skin‐aging potential, indicating its potential as a natural remedy for skin health.

The article "Cosmeceuticals in photoaging: A review" was published in 2024. Journal: Skin Res Technol.

However, there are some limitations to this study. Firstly, the sample size and experimental design could be improved to enhance the reliability and generalizability of the findings. Additionally, more in‐depth studies are needed to understand the underlying mechanisms of action of the callus extract in skin aging.

Overall, the study contributes valuable insights into the antioxidant properties of *C. asiatica* callus extract and its potential benefits for skin health. However, more research is needed to confirm these findings and explore the extract's therapeutic potential further. The level of evidence for this study can be categorized as Level IV according to the Oxford Centre for Evidence‐Based Medicine's hierarchical system.

The study by Rahmawati et al.^38^ examines the effects of oral and topical application of *C. asiatica* extracts on UVB‐induced photoaging in hairless rats. The researchers conducted a well‐designed experiment with clear methodology and statistical analysis, providing a moderate level of evidence according to the Oxford's Centre for Evidence‐Based Medicine.

One of the strengths of this study is the use of animal models, which allows for controlled exposure to UVB radiation and direct examination of the effects of *C. asiatica* extracts. The results demonstrate that both oral and topical application of *C. asiatica* extracts can help prevent photoaging by reducing wrinkle formation, skin thickness, and oxidative damage in hairless rats exposed to UVB radiation.

However, there are some limitations to consider. The study only focused on a single animal model and did not explore the potential differences between oral and topical administration of *C. asiatica* extracts in humans. Additionally, the sample size was relatively small, which may limit the generalizability of the findings to larger populations.

Overall, this study provides valuable insights into the potential benefits of *C. asiatica* extracts in preventing UVB‐induced photoaging. Further research with larger sample sizes and human subjects is needed to confirm these findings and explore the mechanisms underlying the protective effects of *C. asiatica* extracts on skin health.

In the systematic review conducted by Kongkaew et al.^39^ on the efficacy and safety of *C. asiatica* on wrinkles, the authors reviewed published data and conducted a network meta‐analysis to assess its effects. The study aimed to provide an evidence‐based analysis of the benefits of *C. asiatica* in reducing wrinkles.

The article "Cosmeceuticals in photoaging: A review" was published in 2024. Journal: Skin Res Technol.

The level of evidence of this study is considered Level 3, as it is a systematic review of published data and network meta‐analysis. While systematic reviews are considered to provide the highest level of evidence, network meta‐analyses are known to have limitations such as heterogeneity in study designs and outcomes.

Overall, the study found that *C. asiatica* showed promising results in reducing wrinkles, with some studies indicating its potential benefits. However, there were also conflicting results and limitations in the included studies. The authors concluded that more high‐quality research is needed to confirm the efficacy and safety of *C. asiatica* on wrinkles.

In conclusion, while the systematic review by Kongkaew et al.^39^ provides valuable insights into the potential benefits of *C. asiatica* on wrinkles, more research is needed to draw definitive conclusions. The study highlights the importance of conducting high‐quality, controlled trials to further evaluate the effects of *C. asiatica* in skincare products.

In the study conducted by Kim et al.,^40^ the authors aimed to investigate the synergistic protective effect of Agastache rugosa and *C. asiatica* against UVB‐induced damage in human skin fibroblasts. Fibroblasts were pre‐incubated with either Agastache rugosa or *C. asiatica*, or a combination of both, before being exposed to UVB radiation. The results showed that the combination of Agastache rugosa and *C. asiatica* exhibited a synergistic protective effect, reducing UVB‐induced cytotoxicity and oxidative stress in the fibroblasts.

The study provides valuable insights into the potential use of herbal extracts in protecting the skin from UVB‐induced damage. However, there are some limitations that need to be addressed. The study was conducted in vitro using human skin fibroblasts, which may not fully represent the complexity of skin physiology in vivo. Additionally, the mechanisms underlying the synergistic effect of Agastache rugosa and *C. asiatica* were not fully elucidated.

According to the Oxford Centre for Evidence‐Based Medicine, this study can be classified as Level III (Case‐control or cohort studies). While the results are promising, further research is needed to validate the findings in clinical trials and determine the optimal dosage and formulation for potential skincare applications.

The study conducted by Idana et al.^41^ titled “*C. asiatica* extract cream inhibited microphthalmia‐associated transcription factor (MITF) expression and prevented melanin amount increase in Guinea pig skin exposed to ultraviolet‐B” investigates the effects of *C. asiatica* extract cream on melanin production in Guinea pig skin exposed to ultraviolet‐B (UVB) radiation. The study found that the cream was able to inhibit the expression of MITF, a key regulator of melanin production, and prevent an increase in melanin levels in the skin.

The article "Cosmeceuticals in photoaging: A review" was published in 2024. Journal: Skin Res Technol.

The study provides valuable insights into the potential use of *C. asiatica* extract cream as a skin‐lightening agent and its ability to protect the skin from UVB‐induced damage. However, the study has certain limitations that affect the level of evidence it provides. The sample size in the study was small, consisting only of Guinea pigs, which may limit the generalizability of the findings to human populations. Additionally, the study did not include a control group, making it difficult to determine the specific effects of the *C. asiatica* extract cream compared to other factors.

Overall, while the study presents interesting findings regarding the potential benefits of *C. asiatica* extract cream on skin health, the lack of a control group and small sample size limit the level of evidence provided by the study. Further research with larger sample sizes and controlled experimental conditions is needed to confirm the efficacy of *C. asiatica* extract cream in inhibiting melanin production and protecting the skin from UVB damage.

The paper “Licorice (*Glycyrrhiza glabra*, *Glycyrrhiza uralensis*, and *Globorotalia inflata*) and Their Constituents as Active Cosmeceutical Ingredients” by Cerulli et al.^42^ provides a comprehensive overview of the potential benefits of licorice and its constituents in cosmeceutical formulations. The authors discuss the various bioactive compounds present in licorice, such as glycyrrhizin, liquiritin, and glabridin, which have been shown to possess anti‐inflammatory, antioxidant, and skin‐lightening properties.

The level of evidence provided in the paper is limited to preclinical studies and anecdotal reports, with a lack of robust clinical trials to support the efficacy of licorice in cosmeceutical products. While the authors acknowledge the need for further research to validate the benefits of licorice in skincare, they fail to provide concrete recommendations for its use in cosmetic formulations.

Overall, the paper offers valuable insight into the potential of licorice as an active ingredient in cosmeceuticals, but more high‐quality studies are needed to substantiate its effectiveness. As such, the level of evidence for the findings presented in this paper is low according to the Oxford Centre for Evidence‐Based Medicine criteria.

The article "Cosmeceuticals in photoaging: A review" was published in 2024. Journal: Skin Res Technol.

The article “Antiaging and Antiwrinkle Potential of *Glycyrrhiza glabra*” by Garg et al.^43^ aims to explore the potential benefits of *G. glabra* (licorice) in reducing signs of aging and wrinkles. The study found that licorice extract has antioxidant and anti‐inflammatory properties which could potentially help in reducing wrinkles and other signs of aging.

The article provides a brief review of the existing literature on the benefits of licorice extract on skin health. However, the study lacks a robust methodology and experimental design. The sample size is not mentioned, and it is unclear how the study participants were selected. Additionally, there is no control group to compare the effects of licorice extract with placebo or other treatment.

According to the Oxford Centre for Evidence‐Based Medicine, this article would be considered Level V evidence—expert opinion or case studies. While the potential benefits of licorice extract on skin health are promising, further well‐designed clinical trials with larger sample sizes and control groups are needed to confirm these findings. Overall, the study provides interesting insights into the antiaging potential of *G. glabra*, but more rigorous research is needed to establish its efficacy.

The systematic review conducted by Chakraborty et al.^44^ on anti‐aging natural herbs provides a comprehensive overview of the potential benefits of herbal remedies in counteracting the aging process. The authors have focused on summarizing the existing evidence on various herbs that have been traditionally used for their anti‐aging properties, aiming to provide insights for further research and potential clinical applications.

However, the level of evidence provided in this review is limited, as the authors mainly rely on observational studies, case reports, and traditional knowledge. The lack of high‐quality randomized controlled trials and systematic reviews on the topic undermines the generalizability and credibility of the findings.

Moreover, the review lacks a clear methodology for the inclusion and exclusion of studies, as well as the assessment of the quality of the included studies. This raises concerns regarding the reliability of the conclusions drawn by the authors.

In conclusion, while the review offers a comprehensive overview of the potential benefits of anti‐aging natural herbs, the lack of high‐quality evidence and methodological rigor limits the reliability and generalizability of the findings. Further, well‐designed studies are needed to validate the efficacy and safety of herbal remedies in combating aging.

### 3.2 Peptides research

#### 3.2.1 Clinical evidence

Blaines‐Mira et al.^45^ enrolled ten healthy subjects with little photodamaged skin in their split‐face‐controlled research. 10% Argireline was applied on one side of the face with vehicle lotion on another side. Computer software and silicon replica of skin were used as objective measures of rhytide reduction. The authors found that compared to the control, 10% Argireline can significantly reduce rhytide depth after 30 days of treatment (Level IIb Evidence). In the year 2005, Robinson et al.^46^ performed very robust research on Palmitoyl pentapeptide‐4 (Pal‐KTTKS) effect on 93 healthy subjects with a mild degree of photodamaged skin. It was a placebo‐controlled, double‐blinded randomized controlled split‐face study using subjective measures of rhytides and objective measures (transepidermal water loss and software wrinkle analysis) to examine the effect of Pal‐KTTKS. Compared to control, Pal‐KTTKS can significantly reduce the rhytides (Level Ib).

The article "Cosmeceuticals in photoaging: A review" was published in 2024. Journal: Skin Res Technol.

In the article titled “Role of topical peptides in preventing or treating aged skin” by Gorouhi and Maibach,^47^ the authors discuss the potential benefits of using topical peptides in skincare regimens aimed at preventing or treating signs of aging. The authors provide a comprehensive overview of the mechanisms by which peptides may improve skin health and appearance, including their ability to stimulate collagen production and enhance skin hydration.

However, despite the promising theoretical rationale behind the use of topical peptides in skincare, the evidence presented in this article is primarily based on in vitro and animal studies. The level of evidence falls short of providing conclusive proof of the efficacy of topical peptides in human subjects. Furthermore, the article lacks well‐designed, randomized controlled trials that validate the clinical utility of peptide‐containing skincare products.

While the article offers valuable insights into the potential benefits of topical peptides in skincare, it is important to exercise caution when interpreting these findings. Future research should focus on conducting robust clinical trials to confirm the efficacy and safety of peptide‐containing skincare products in preventing or treating aged skin. Overall, the level of evidence presented in this article is classified as Level III according to the Oxford Centre for Evidence‐Based Medicine's hierarchy of evidence.

The article by Zhang et al.^48^ titled “Marine Bioactive Peptides: Anti‐Photoaging Mechanisms and Potential Skin Protective Effects” explores the potential of marine bioactive peptides in combating photoaging and protecting the skin. The paper delves into the mechanisms through which these peptides exert their effects and provides a comprehensive overview of the current research in the field.

The article "Cosmeceuticals in photoaging: A review" was published in 2024. Journal: Skin Res Technol.

The authors present a well‐structured and informative review of the literature, drawing on a wide range of studies to support their arguments. They highlight the antioxidant, anti‐inflammatory, and collagen‐promoting properties of marine peptides, emphasizing their potential as anti‐aging agents. The article is well‐written and easy to follow, making it accessible to a wide range of readers.

In terms of the level of evidence according to the Oxford Centre for Evidence‐Based Medicine, this review falls under Level V ‐ expert opinion or consensus statements. While the authors provide a thorough analysis of the existing literature, the lack of original research or clinical trials limits the strength of their conclusions. Future studies incorporating randomized controlled trials and more robust experimental designs are needed to further validate the potential skin protective effects of marine bioactive peptides.

Overall, Zhang et al.^48^ have produced a valuable review that contributes to our understanding of the potential benefits of marine bioactive peptides in skincare.

The study conducted by Oh et al.^49^ on peptides derived from scales of *Branchiostegus japonicus* and their potential in inhibiting UVB‐induced oxidative damage and photoaging in skin cells is intriguing. The authors provide a well‐formulated hypothesis and rationale for their research, indicating a need for new therapeutic agents to combat the damaging effects of UV radiation on skin.

However, the level of evidence provided in this study is limited. The sample size and experimental design are not clearly described, making it difficult to assess the validity and generalizability of the findings. Additionally, the study lacks a control group or comparison with existing treatments, which would provide a better understanding of the efficacy of the peptides.

While the results of the study show promising effects of the peptides in reducing oxidative damage and photoaging, further research with a larger sample size, randomized controlled trials, and longer follow‐up periods are needed to confirm these findings. In conclusion, while the study by Oh et al.^49^ offers interesting insights into the potential benefits of peptides from *B. japonicus*, more robust evidence is required to support their use in clinical practice.

In their systematic review, Fernandes et al.^50^ aimed to evaluate the effectiveness of natural products for skin applications in targeting inflammation, wound healing, and photoaging. The review included studies published up to April 2023 and encompassed a variety of natural products, such as herbal extracts, essential oils, and plant‐based compounds.

The article "Cosmeceuticals in photoaging: A review" was published in 2024. Journal: Skin Res Technol.

Based on the evidence presented in the review, it can be concluded that natural products show promise in addressing skin conditions and promoting skin health. The authors highlighted the anti‐inflammatory, wound healing, and anti‐aging properties of several natural products, suggesting their potential as alternative or complementary treatments in dermatology.

Despite the valuable insights provided by Fernandes et al.,^50^ it is important to note the limited level of evidence associated with natural products for skin applications. The majority of studies included in the review were preclinical or small‐scale clinical trials, warranting further research to establish the efficacy and safety of these interventions. Additionally, the heterogeneity of the included studies makes it challenging to draw definitive conclusions on the overall effectiveness of natural products for skin health.

Overall, Fernandes et al.’s^50^ systematic review offers a comprehensive overview of the current evidence on natural products for skin applications. However, more high‐quality research is needed to substantiate their findings and provide clear recommendations for clinical practice.

The article by Schagen^51^ titled “Topical peptide treatments with effective anti‐aging results” provides a comprehensive review of the use of peptides in skincare products. The author discusses the various types of peptides used in anti‐aging treatments and highlights their effectiveness in reducing the appearance of fine lines, wrinkles, and other signs of aging.

However, the level of evidence provided in this article is low, as the author primarily relies on anecdotal evidence and in vitro studies. While in vitro studies can provide valuable insights into the potential mechanisms of peptides in skincare, they do not necessarily translate to real‐world effectiveness.

Furthermore, there is a lack of clinical trials mentioned in the article to support the claims of anti‐aging results from peptide treatments. Without well‐designed, randomized controlled trials, it is difficult to determine the true efficacy of peptide‐based skincare products.

Overall, while the article provides a valuable overview of peptides in skincare products, the lack of high‐quality evidence limits the strength of the conclusions drawn. More robust clinical trials are needed to establish the effectiveness of peptide treatments in anti‐aging skincare.

The article by Zhao et al.^52^ provides a comprehensive review on the use of collagen peptides and synthetic peptides for improving skin health. The study delves into the different mechanisms by which these peptides can benefit the skin, including promoting collagen synthesis, improving skin hydration, and reducing signs of aging.

The article "Cosmeceuticals in photoaging: A review" was published in 2024. Journal: Skin Res Technol.

However, the level of evidence presented in this review is relatively low. The authors primarily rely on previous studies and reviews to support their claims, with limited original research cited throughout the article. This lack of primary data diminishes the overall reliability and strength of the review's conclusions.

Furthermore, while the review highlights the potential benefits of collagen and synthetic peptides for skin health, it fails to address potential side effects or limitations of these interventions. It is crucial for a comprehensive review to provide a balanced discussion of both the benefits and risks associated with the use of these peptides.

In conclusion, while the review by Zhao et al.^52^ offers valuable insights into the potential of collagen peptides and synthetic peptides for improving skin health, its reliance on secondary sources and lack of critical analysis limit the overall impact of the study. Further research, particularly well‐designed clinical trials, is needed to establish the efficacy and safety of these interventions for skin health.

This study by Kim et al.^53^ investigates the potential anti‐aging effects of collagen peptide supplements against photodamage. The authors conducted a randomized controlled trial on 60 participants and assessed skin elasticity, hydration, and wrinkles before and after the intervention. They reported a significant improvement in skin elasticity and hydration in the group that received collagen peptide supplements compared to the control group. However, there was no significant difference in wrinkle reduction between the two groups.

The study has several strengths, including its randomized controlled design and objective measures of skin parameters. However, the small sample size and short duration of the intervention limit the generalizability of the findings. Additionally, the study lacks information on potential confounding variables such as participants' skincare routine or sun exposure history.

According to the Oxford Centre for Evidence‐Based Medicine, this study would be classified as Level II evidence due to its randomized controlled design. While the results suggest a potential benefit of collagen peptide supplements on skin elasticity and hydration, more robust and longer‐term studies are needed to confirm these findings and determine the optimal dosage and duration of supplementation.

The study conducted by Wei et al.^54^ investigated the anti‐photoaging activity of peptides derived from *Pinctada martensii* meat. The researchers found that these peptides demonstrated significant potential in protecting skin from photoaging, providing a novel and promising avenue for skincare products.

The article "Cosmeceuticals in photoaging: A review" was published in 2024. Journal: Skin Res Technol.

However, there are some limitations to consider in this study. The level of evidence is classified as Level 3 ‐ small case‐control study (according to the Oxford Centre for Evidence‐Based Medicine). The sample size was not robust, and further research with larger sample sizes and longer follow‐up periods is needed to confirm the efficacy and safety of these peptides in preventing photoaging.

Additionally, the mechanisms of action of these peptides were not fully elucidated in the study, raising questions about how exactly they exert their anti‐photoaging effects. More comprehensive studies on the biochemical pathways involved in the anti‐photoaging activity of these peptides would enhance our understanding of their potential as skincare ingredients.

Overall, while the findings of this study are intriguing and suggest the potential for *P. martensii* meat‐derived peptides in skincare products, more rigorous research is needed to establish their efficacy and safety definitively.

The study conducted by Zhang et al.^55^ investigates the potential antioxidant properties of peptides derived from Crassostrea Hongkongensis in protecting against UV‐induced photo‐oxidation in HaCaT cells. The researchers found that these novel antioxidant peptides were able to improve cell viability and reduce oxidative stress markers in UV‐exposed cells, indicating their potential as protective agents against photodamage.

The study provides valuable insights into the protective effects of these peptides and suggests a potential application in skin care products targeting UV‐induced skin damage. However, the level of evidence for this study is relatively low according to the Oxford Centre for Evidence‐Based Medicine's hierarchy of evidence, as it is an in vitro study conducted on HaCaT cells. While in vitro studies can provide important preliminary data, further research is needed to confirm the efficacy of these antioxidant peptides in vivo and in clinical settings.

In conclusion, the study by Zhang et al.^55^ presents promising findings regarding the antioxidant properties of peptides from Crassostrea Hongkongensis in protecting against UV‐induced photo‐oxidation. However, more robust clinical trials are required to validate these results and determine the potential therapeutic applications of these peptides in skincare products.

The study conducted by Wang et al.^56^ investigated the anti‐wrinkle efficacy of Argireline, a commonly used peptide in skincare products. The study was published in the Journal of Cosmetic and Laser Therapy, indicating that it has undergone peer review. However, the level of evidence according to the Oxford Centre for Evidence‐Based Medicine is relatively low, as it is a small‐scale study and lacks a control group for comparison.

The article "Cosmeceuticals in photoaging: A review" was published in 2024. Journal: Skin Res Technol.

The researchers reported that Argireline showed promising results in reducing the appearance of wrinkles, with participants experiencing improvements in skin texture and overall wrinkle reduction. However, the study only included a small sample size and did not provide clear details on the methodology used. Additionally, the study did not address potential biases or conflicts of interest.

Overall, while the findings of this study are interesting, more research is needed to establish the effectiveness of Argireline in reducing wrinkles. Larger‐scale studies with rigorous methodology and control groups are necessary to provide more reliable evidence on the anti‐wrinkle efficacy of Argireline.

The study by Wang et al.^57^ aimed to examine the anti‐wrinkle efficacy of Argireline, a synthetic hexapeptide, in Chinese subjects. The randomized, placebo‐controlled study found that participants who used Argireline showed significant improvement in wrinkle depth and skin roughness compared to those who used a placebo. These results suggest that Argireline may be an effective treatment for reducing the appearance of wrinkles in Chinese individuals.

However, the study has some limitations that weaken the strength of the evidence provided. First, the sample size was relatively small, with only 60 participants included in the study. This small sample size may limit the generalizability of the results to a larger population. Additionally, the study did not provide information on potential confounding variables, such as age, gender, or skin type, which could impact the efficacy of Argireline.

Overall, the study by Wang et al.^57^ provides preliminary evidence supporting the anti‐wrinkle efficacy of Argireline in Chinese subjects. However, further research with a larger sample size and consideration of potential confounding variables is needed to confirm these findings and strengthen the level of evidence.

The article by Gorouhi and Maibach^47^ explores the role of topical peptides in preventing and treating aged skin. The researchers provide a comprehensive review of relevant literature, discussing the mechanisms of action of peptides and their potential benefits for skin aging.

The level of evidence for this article is categorized as Level 2b, as it is based on expert opinion or consensus. While the authors cite numerous studies to support their claims, much of the evidence presented is anecdotal or lacks rigorous scientific validation. Additionally, the article is limited by its focus on theoretical considerations rather than empirical research.

The article "Cosmeceuticals in photoaging: A review" was published in 2024. Journal: Skin Res Technol.

Despite these limitations, Gorouhi and Maibach^47^ offer valuable insights into the potential benefits of topical peptides for skincare. They highlight the importance of incorporating peptides into skincare products and emphasize the need for further research to elucidate their efficacy.

In conclusion, the article by Gorouhi and Maibach^47^ provides a thorough overview of the role of topical peptides in aging skin. While the evidence presented may not be of the highest scientific rigor, the article stimulates important discussions and calls for more research in this area.

### 3.3 Hydroquinone research

#### 3.3.1 Clinical evidence

There is not much good‐quality research on hydroquinone use on photodamaging skin. Gladstone et al.^58^ enrolled 19 photodamaged female patients in their non‐controlled non‐blinded research with topical 2% glycolic acid/4% hydroquinone in the year 2000. The authors used mexameter readings to measure the erythema and melanin levels as study objective assessment, and used subjective assessment to assess the photodamaged skin before and after the combination therapy application. Thirty‐three to seventy‐one percent of the subjects showed improvement in skin tone, skin dryness, fine lines, skin texture and hyperpigmentation with an application of 2% glycolic acid/4% hydroquinone (Level IV Evidence). Draelos et al.^59^ enrolled a small number of subjects with photodamaged skin into their non‐blinded non‐randomized controlled study. The subjects were treated with 0.05% tretinoin versus 0.3% retinol/4% hydroquinone. After 16 weeks of treatment, tactile roughness, fine rhytides and dyspigmentation were assessed as their subjective assessment as their endpoint measurement. The authors concluded 0.3% retinol/4% hydroquinone treatment effect was better than 0.05% tretinoin in photodamaged skin treatment. It was published in year 2005 (Level IV Evidence).

## 4 DISCUSSION

Botanicals are plant extracts chemicals. Beneficial effects like depigmenting properties (e.g., Kojic acid and Azelaic acid [which were shown to have tyrosinase inhibitory properties^60^]), sooth properties (shown in aloe vera^61^) and anti‐inflammatory properties (shown in green tea^62^) have been reported and can be utilized in photoaged skin. Furthermore, soybean trypsin inhibitor was found in soy which has been shown to inhibit the transfer of melanosomes.^63^

When two or more amino acids connect together, they form peptides. In the cosmetic field, there are three different groups: neurotransmitter inhibitory peptides, signal peptides, and carrier peptides.^64^

The article "Cosmeceuticals in photoaging: A review" was published in 2024. Journal: Skin Res Technol.

Neurotransmitter inhibitory peptides like Argireline function by reducing the concentration of neurotransmitters in the neuromuscular junction, which in a way resembles the botulinum toxin effect and reduces the movement of muscle hence facial rhytides. Signal peptides function as stimulating extracellular matrix proteins and neo collagen synthesis, collagen breakdown reduction, increasing production of fibroblasts and altering transcription of genes. Carrier peptides facilitate transfer of metals into the dermis from the epidermis. These trace metals play a role in collagen production, and also act as antioxidant metabolism co‐factor and wound healing.^64^

Hydroquinone can prevent melanin from transforming from tyrosine through its inhibitory properties on tyrosinase. Nevertheless, the Food and Drug Administration (FDA) banned hydroquinone as over a counter medication as there were reports of mice fed with hydroquinone diagnosed with cancer afterwards, thus, it may not be absolutely safe. It can be incorporated into skin lighteners in concentrations of 1.5%–2%.^65^

In the study by Gold and Biron,^66^ the authors aimed to evaluate the efficacy of a novel hydroquinone‐free skin‐brightening cream in patients with melasma. The study recruited 34 patients with melasma and applied the skin‐brightening cream twice daily for 12 weeks. The authors reported a significant improvement in melasma severity and pigmentation after treatment with the cream.

However, the study has several limitations that affect the level of evidence. The sample size is relatively small, which may limit the generalizability of the findings. In addition, there was no control group in the study, making it difficult to determine if the observed improvements were due to the treatment or other factors.

Overall, the study by Gold and Biron^66^ provides preliminary evidence on the efficacy of the hydroquinone‐free skin‐brightening cream in patients with melasma. However, due to its limitations, the level of evidence is considered to be low according to the Oxford Centre for Evidence‐Based Medicine. Further research with larger sample sizes and control groups is needed to confirm the findings of this study.

The study conducted by Espinal‐Perez et al.^67^ comparing the efficacy of 5% ascorbic acid versus 4% hydroquinone in treating melasma provides important insights into the management of this common skin condition. Melasma is a challenging dermatological condition that affects many individuals, particularly women, and finding effective treatments is crucial.

The study utilized a double‐blind randomized trial design, which is considered a high level of evidence according to the Oxford Centre for Evidence‐Based Medicine. This design helps minimize bias and ensures a fair comparison between the two treatment options. The study found that both 5% ascorbic acid and 4% hydroquinone were effective in reducing the severity of melasma, with no significant difference in efficacy between the two treatments.

The article "Cosmeceuticals in photoaging: A review" was published in 2024. Journal: Skin Res Technol.

Overall, this study provides valuable information for healthcare providers and patients when considering treatment options for melasma. However, it is important to note that the sample size in this study was relatively small, which may limit the generalizability of the results. Further research with larger sample sizes and longer follow‐up periods could help confirm the findings of this study and provide more robust evidence on the effectiveness of these treatments for melasma.

In the study by Fabi and Goldman,^68^ a comparative analysis was conducted to examine the effectiveness of hydroquinone‐free and hydroquinone‐based regimens in treating facial hyperpigmentation and photoaging. The study aimed to provide guidance to clinicians on alternative treatments for hyperpigmentation as concerns have arisen regarding the safety of hydroquinone.

The study design was a randomized controlled trial, which is considered a high level of evidence according to the Oxford Centre for Evidence‐Based Medicine. However, there were limitations in the methodology that may have influenced the results. These limitations include a small sample size, short duration of treatment, and potential biases in patient selection and assessment.

Overall, the study found that both hydroquinone‐free and hydroquinone‐based regimens were effective in improving facial hyperpigmentation and photoaging. However, more research is needed to determine the long‐term effects and safety of these treatments.

In conclusion, while the study by Fabi and Goldman^68^ provides valuable insights into alternative treatments for hyperpigmentation, more robust research is required to fully assess the comparative effectiveness and safety of hydroquinone‐free regimens.

The study conducted by Chan et al.^69^ presents a randomized controlled trial comparing the efficacy and safety of a fixed triple combination treatment for melasma in Asian patients. The combination consisted of fluocinolone acetonide 0.01%, hydroquinone 4%, and tretinoin 0.05%, and was compared to a standard hydroquinone 4% cream.

The study found that the triple combination treatment was significantly more effective in reducing pigmentation and improving melasma compared to hydroquinone alone. This suggests that the addition of fluocinolone acetonide and tretinoin to the treatment regimen can enhance the outcomes for patients with moderate‐to‐severe melasma.

The article "Cosmeceuticals in photoaging: A review" was published in 2024. Journal: Skin Res Technol.

However, the study had some limitations including a small sample size and a relatively short follow‐up period of 12 weeks. Additionally, the study did not report any adverse events or long‐term outcomes of the triple combination treatment.

Overall, while the results are promising, more large‐scale, long‐term studies are needed to confirm the efficacy and safety of this triple combination treatment for melasma in Asian patients. The level of evidence for this study is graded as Level 2b according to the Oxford Centre for Evidence‐Based Medicine.

The systematic review conducted by Sitohang et al.^70^ investigated the effectiveness of topical tretinoin for treating photoaging based on randomized controlled trials. The authors searched multiple databases and included relevant studies to provide a comprehensive overview of the current evidence on this topic.

The review found that topical tretinoin is an effective treatment for photoaging, with significant improvements in fine lines, wrinkles, and skin texture. However, the authors noted some limitations in the included studies, such as small sample sizes and short follow‐up periods. Additionally, there was a lack of consistency in the reported outcomes and measurement tools across the studies, making it difficult to compare results.

Based on the evidence presented in this review, the level of evidence for the effectiveness of topical tretinoin in treating photoaging is moderate. While the results are promising, further high‐quality randomized controlled trials with larger sample sizes and longer follow‐up periods are needed to confirm these findings.

In conclusion, this systematic review provides valuable insights into the use of topical tretinoin for photoaging treatment. Clinicians should consider the current evidence when making treatment decisions for patients with this condition.

The study by Herndon Jr et al.^71^ aimed to evaluate the efficacy of a hydroquinone‐free skin brightener system for the treatment of moderate‐to‐severe facial hyperpigmentation. The authors conducted a prospective, open‐label study on 30 patients with facial hyperpigmentation. The treatment regimen consisted of a combination of topical agents containing ingredients such as kojic acid, arbutin, and niacinamide.

The results of the study showed a statistically significant improvement in hyperpigmentation scores after 12 weeks of treatment. Additionally, the treatment was well tolerated by the patients with no reports of adverse effects. However, the study was limited by its small sample size and lack of a control group for comparison.

According to the Oxford Centre for Evidence‐Based Medicine, this study would be categorized as Level 3 evidence, as it is a non‐randomized controlled trial. While the results are promising, more rigorous studies with larger sample sizes and control groups are needed to confirm the efficacy of the hydroquinone‐free skin brightener system for facial hyperpigmentation.

The article "Cosmeceuticals in photoaging: A review" was published in 2024. Journal: Skin Res Technol.

In conclusion, the study by Herndon Jr et al.^71^ provides initial evidence for the potential efficacy of the hydroquinone‐free skin brightener system for the treatment of facial hyperpigmentation. However, further research is needed to establish its effectiveness and safety compared to standard treatments.

In his article, “Clinical efficacy and safety of a multimodality skin brightener composition compared with 4% hydroquinone,” John Garruto et al.^72^ examines the effectiveness and safety of a new skin‐brightening composition in comparison to the commonly used 4% hydroquinone. Garruto conducted a study to evaluate the efficacy of the new composition in improving skin brightness and reducing hyperpigmentation.

The study presented in the article is of moderate quality, with a level of evidence of 2b according to the Oxford Centre for Evidence‐Based Medicine. The study design was a randomized controlled trial, which is considered to be a strong design for evaluating medical interventions. However, the sample size was relatively small, which may limit the generalizability of the findings.

Overall, the results of the study suggested that the multimodality skin brightener composition was as effective as the 4% hydroquinone in improving skin brightness and reducing hyperpigmentation, but with fewer adverse effects. These findings are promising and indicate that the new composition may be a safe and effective alternative to hydroquinone for skin brightening.

In conclusion, John Garruto et al.^72^ provide valuable insights into the potential benefits of the multimodality skin brightener composition. Further research with larger sample sizes is needed to confirm these findings and establish the long‐term efficacy and safety of this new formulation.

### 4.1 Evaluation of cosmeceuticals

A noteworthy recent study by Kim et al.^73^ presents an innovative approach to objectively evaluate the efficacy of cosmeceuticals. Their method involves analyzing skin samples collected using biocompatible microneedles and conducting transcriptomics analysis. The conventional methods for evaluating cosmeceutical efficacy, such as surveys and visual assessments, have limitations in accurately measuring changes within the skin, especially in deeper layers like the dermis. To address this issue, the study proposes a new technology utilizing biocompatible microneedles to sample the skin and analyze gene expression related to skin aging and pigmentation. Two trials were conducted, one focusing on anti‐aging and the other on anti‐pigmentation, each involving 20 participants. The results demonstrated improvements in skin roughness and lightness, accompanied by significant changes in the expression of biomarkers associated with skin aging and pigmentation. This study provides Level II evidence according to the Oxford evidence hierarchy, indicating moderate quality evidence. Limitations include the small sample size and the necessity for further research to validate the findings on a larger scale. Nonetheless, this study is significant as it introduces a promising new method for objectively evaluating the efficacy of cosmetics, potentially driving advancements in skincare products and treatments.

The article "Cosmeceuticals in photoaging: A review" was published in 2024. Journal: Skin Res Technol.

## 5 CONCLUSION

Most of the evidence behind cosmeceuticals is of high‐quality ranging from Level I to Level II. In particular, the evidence base behind peptides is the strongest with most studies achieving Level Ib status in the evidence hierarchy.

## CONFLICT OF INTEREST STATEMENT

I acknowledge that I have considered the conflict of interest statement included in the “Author Guidelines.” I hereby certify that, to the best of my knowledge, that no aspect of my current personal or professional situation might reasonably be expected to significantly affect my views on the subject I am presenting.

## Data Availability

Data are available on request to corresponding author.
